# LncRNA PCGEM1 induces proliferation and migration in non-small cell lung cancer cells through modulating the miR-590-3p/SOX11 axis

**DOI:** 10.1186/s12890-021-01600-9

**Published:** 2021-07-14

**Authors:** Huanshun Wen, Hongxiang Feng, Qianli Ma, Chaoyang Liang

**Affiliations:** Department of Thoracic Surgery, China-Japan Friendship Hospital, No. 2 Yinghua East Street, Chaoyang District, Beijing, 100029 China

**Keywords:** Non-small cell lung cancer, PCGEM1, miR-590-3p, SOX11

## Abstract

**Background:**

Non-small cell lung cancer (NSCLC) is one of the most prevalent cancers. As reported, long non-coding RNAs (lncRNAs) induce various biological behaviors in cancers. LncRNA PCGEM1 prostate-specific transcript (PCGEM1) is reported to exert carcinogenic effect on certain cancers. Our research aimed to explore the role of PCGEM1 in NSCLC.

**Methods:**

We enrolled forty NSCLC patients to explore PCGEM1 expression in clinical NSCLC tissues. Colony formation assay, CCK-8, Transwell assay were conducted to reveal cell proliferation, viability, migration and invasion. Luciferase reporter assay, RNA pull down, and RIP assay were performed to investigate the downstream axis of PCGEM1.

**Results:**

PCGEM1 was significantly upregulated in NSCLC cells and tissues. Subsequently, *in vitro* loss-of-function experiments illustrated the carcinogenic role of PCGEM1 in NSCLC through promoting viability, proliferation, migration, and invasion. MiR-590-3p was confirmed to be a downstream gene of PCGEM1. Furthermore, SRY-box transcription factor 11 (SOX11) was verified to be a target of miR-590-3p. Additionally, rescue experiments indicated that miR-590-3p inhibitor or pcDNA3.1/SOX11 rescued the impacts of downregulated PCGEM1 on NSCLC cell proliferation, viability, migration and invasion.

**Conclusions:**

LncRNA PCGEM1 aggravated proliferative and migrative abilities in NSCLC via the miR-590-3p/SOX11 axis.

**Supplementary Information:**

The online version contains supplementary material available at 10.1186/s12890-021-01600-9.

## Background

Nowadays, non-small cell lung cancer (NSCLC) is one of the most common malignancies worldwide and is a main reason for the cancer-related mortalities worldwide [1–3], accounting for larger proportion of death causes than breast, prostate and colon cancers combined [4, 5]. The incidence of NSCLC has shown a significant rise in recent years [3, 6]. Despite significant progress in the diagnosis and treatment of NSCLC, five-year survival rates are 14−49% for patients with stage I to stage III NSCLC and are lower than 5% for patients with stage IIIB/IV NSCLC [7]. Therefore, it is urgent to figure out the potential biomarker of treatment for patients with NSCLC.

Over recent years, most newly discovered transcriptomes are long non-coding RNAs (lncRNAs) that are heterogeneous and uncharacterized [8]. By transcriptional and post-transcriptional mediation, abnormal expression of lncRNA might cause proliferation and migration of cells [9]. A principal theme of lncRNA biology appears to form networks that interact with microRNAs (miRNAs) [8]. As reported, lncRNAs function to be the negative modulators of their downstream miRNA molecules [8]. For example, SOX2OT contributes to hepatocellular carcinoma progression via sponging miR-122-5p [10]. LINC00520 acts as an oncogene in malignant melanoma through interacting with miR-125b-5p [11]. Furthermore, PITPNA-AS1 aggravates cervical cancer progression via acting as an miR-876-5p sponge [12]. PCGEM1 prostate-specific transcript (PCGEM1), also termed LINC00071, NCRNA00071, or PCAT9, is encoded on 2q32 and is one of the earliest lncRNAs described in prostate cancer [13]. PCGEM1 is located at chr2: 193,614,571−193,641,625 at the length of 27,055 bp and its orientation is plus strand. Studies have revealed that PCGEM1 acts as a tumor promoter in renal carcinoma [14], cervical cancer [15], and gastric cancer [16] by facilitating cancer cell proliferation and migration. We hypothesized that PCGEM1 functions as an oncogene in NSCLC by promoting NSCLC cell proliferation and migration.

Our report studied the biological role and regulatory mode of PCGEM1 in NSCLC. It was concluded that lncRNA PCGEM1 facilitated cell proliferation, migration, and invasion in NSCLC via modulating the miR-590-3p/SOX11 axis. The findings indicated that PCGEM1 could provide a new vision for NSCLC diagnosis.

## Materials and methods

### Tissue samples

Forty pairs of NSCLC tissues and adjacent noncancerous tissues were obtained from NSCLC patients from China-Japan Friendship Hospital (Beijing, China) after obtaining the participants’ informed consents and the approval from the Ethics Committee of the China-Japan Friendship Hospital (Beijing, China). The collected tissues were immediately frozen in liquid nitrogen, and were subsequently stored at -80℃ for the following research. None of patients had received anticancer treatments before the surgery.

### Cell lines

NSCLC cell lines, A549, H1299, H460, H1975, an immortalized human lung epithelial cell line, BEAS-2B, and a human kidney cell line, human embryonic kidney 293T (HEK293T), were provided by the American Type Culture Collection (ATCC, USA). In brief, all cells were cultured in Dulbecco’s modified Eagle’s medium (DMEM; Gibco, Waltham, MA, USA) supplemented with 10% fetal bovine serum (FBS, Wolcavi, Beijing, China), 100 U/ml penicillin (Sigma-Aldrich, USA), and 100 mg/mL streptomycin (Sigma-Aldrich, USA) in the specific medium under the environment of 37 °C with 5% of CO_2_.

### Cell transfection

The sh-RNA sequences targeting lncRNA PCGEM1 (#1: 5′-AUGAGGGCCCAUCUACAAAUU-3′; #2: 5′-AGUGUGAAAUCUAUUAGUCUU-3′) and sh-NC (5′-AUGGACACCAUCUAGAGCAUU-3′) were purchased from Genepharma (Shanghai, China). To produce pcDNA3.1/SOX11, the sequence of SOX11 (mRNA) was synthesized and subcloned into pcDNA3.1 (Invitrogen, Carlsbad, USA) plasmid. Moreover, NSCLC cells or HEK293T cells were transfected with miR-590-3p mimics (inhibitor) or NC mimics (inhibitor) by Lipofectamine 2000. MiR-590-3p mimics (inhibitor) and NC mimics (inhibitor) were both supplied by GenePharma (Shanghai, China). Transfection efficiency was determined by RT-qPCR.

### Real-time quantitative polymerase chain reaction (RT-qPCR)

Total RNAs were extracted from frozen tissue samples or cells using TRIzol reagent kits (Huamai, Beijing, China) based on the manufacturer’s guidance. Total RNAs were reverse transcribed into complementary DNA (cDNA) with PrimeScript RT reagent kits (RRO36A, Takara Biotechnology Ltd., Dalian, Liaoning, China). A SYBR® Premix Ex TaqTM II reagent kit (RR820A, Takara) was utilized to perform RT-qPCR with an ABI7500 real-time qPCR system (7500, ABI Company, Oyster Bay, NY, USA). Glyceraldehyde-3-phosphate dehydrogenase (GAPDH) and U6 were utilized as internal references. U6 was treated as the internal reference for miR-590-3p. GAPDH was used as an internal reference for PCGEM1 and SOX11. The relative RNA expression quantification was calculated with the 2^−△△CT^ method. Relative primer sequences are listed as follows:

- PCGEM1, Forward: 5′-AAACAAAGGTGCCTTTGCC-3′,
  Reverse: 5′-CCCTCAGAAATCTCAGGGC-3′;
- MiR-590-3p, Forward: 5′-TAATTTTATGTATAAGCTAGTCCGCG-3′,
  Reverse: 5′-CTCTACAGCTATATTGCCAGCCAC-3′;
- MiR-3127-5p, Forward: 5′-ATCAGGGCTTGTGGAATGG-3′,
  Reverse: 5′-CTCTACAGCTATATTGCCAGCCAC-3′;
- MiR-548ar-3p, Forward: 5′-TAAAACTGCAGTTATTTTTGCGG-3′,
  Reverse: 5′-CTCTACAGCTATATTGCCAGCCAC-3′;
- MiR-548az-3p, Forward: 5′-AAAAACTGCAATCACTTTTGCG-3′,
  Reverse: 5′-CTCTACAGCTATATTGCCAGCCAC-3′;
- MiR-548e-3p, Forward: 5′-AAAAACTGAGACTACTTTTGCACCG-3′,
  Reverse: 5′-CTCTACAGCTATATTGCCAGCCAC-3′;
- U6, Forward: 5′-ATACAGAGAAAGTTAGCACGG-3′,
  Reverse: 5′-GGAATGCTTCAAAGAGTTGTG-3′.
- SOX11, Forward: 5′-ACGCAGGAAGATCATGGAG-3′,
  Reverse: 5′-CAGCCTCTTGGAGATCTCG-3′;
- LARP4, Forward: 5′-AGTAACTCATGGAACTGAAAGC-3′,
  Reverse: 5′-GAGAGCTCTGCATTACCCT-3′;
- TOB1, Forward: 5′-CTCTGTCCTCTGTCCTCAG-3′,
  Reverse: 5′-ATGTTGACACGTCTCCTGG-3′;
- WASL, Forward: 5′-CTATTGTGGGAACAAGAGCT-3′,
  Reverse: 5′-CTTGACAAGTATCTCCAGCA-3′;
- RC3H2, Forward: 5′-AAGTGGAGGTAAAGGTGTAGC-3′,
  Reverse: 5′-TTTACAAGTGTCACCAGTTTCC-3′;
- ZNF207, Forward: 5′-AGGTATGATGCCACCACAG-3′,
  Reverse: 5′-ACCACCATACTGACCATGAG-3′;
- ACVR2A, Forward: 5′-GCTGTGAGGGCAATATGTG-3′,
  Reverse: 5′-TAACTGGATTTGAAGTGGGCT-3′;
- GAPDH, Forward: 5′-TCATTTCCTGGTATGACAACGA-3′,
  Reverse: 5′-GTCTTACTCCTTGGAGGCC-3′.

### CCK-8 assay

Cell viability in response to PCGEM1 knockdown was measured with a Cell Counting Kit-8 (CCK-8; Dojindo Molecular Technologies, Inc., Kyushu, Japan) following the manufacturer’s guidance. The cells were seeded into 96-well plates (1 × 10^3^ cells/well) in triplicate and measured at days 1, 2, 3, 3, 5. Next, CCK-8 reagent was added, and the cells were incubated for further 2 h at 37 °C. The chromogenic reaction was allowed in a culture incubator for 4 h. The absorbance values were finally determined at 450 nm with a microplate reader (SAFAS Xenius XL, Ruixuan, Shanghai, China).

### Colony formation assay

The colony formation assay was utilized to access the cell proliferation. Transfected cells were diluted and seeded onto 6-well plates at the density of approximately 1 × 10^3^ cells/well. Transfected cells were maintained in DMEM containing 10% FBS, which was replaced every 3 days. Afterward, cells were then cultured at 37 °C for 2 weeks and fixed with methanol and stained with 0.1% crystal violet (Beyotime, Shanghai) for 30 min when colonies were visible. The plates were photographed, and the number of colonies was counted after 48 h.

### Transwell assay

Transwell assay was performed with Transwell chambers (8 μm diameter; Corning Inc., Corning, NY, USA). Transfected cells at a density of 1 × 10^5^ cells/well were plated on upper chambers which were coated without Matrigel and contained serum-free DMEM. DMEM containing 10% FBS was added to the lower chamber. After incubation for 48 h, the cells were harvested, washed with phosphate‐buffered saline (PBS), and resuspended in DMEM without FBS. At 24 h after inoculation, nonmigratory cells were gently removed, and the migratory cells were fixed with 100% methanol, stained with 0.5% crystal violet, washed with PBS, and imaged using an inverted microscope (Olympus Corporation, Tokyo, Japan). The invasion assay was performed like the migration assay except that the chamber was precoated with Matrigel. The migration and invasion abilities were measured through counting the migrated and invaded cells, respectively. Migrated and invaded cells were observed under a light microscope and counted using ImageJ v1.46 software.

### Western blot

Total proteins in cells were extracted with RIPA lysis buffer containing protease and phosphatase inhibitors (Roche, Shanghai, China). Protein concentration was detected by a bicinchoninic acid kit. Then the cell protein lysates were separated by 10% of sodium dodecyl sulfate-polyacrylamide gel electrophoresis, shifted to a polyvinylidene fluoride membrane. Next, membranes were blocked with 5% skim milk powder at room temperature for 1 h and incubated with the primary antibodies including anti-E-cadherin, anti-N-cadherin and anti-GAPDH at 4 °C overnight. All antibodies were purchased from Proteintech (Rosemont, IL, USA). Then the membranes were washed with Tris-buffered saline Tween-20 and further incubated with the horseradish peroxidase-conjugated secondary antibody at room temperature for 1 h. Proteins on the membrane were visualized by enhanced chemiluminescence detection kits (Amersham Pharmacia Biotech, UK) and Bio-Rad image analysis system (Bio-Rad Laboratories, Inc. CA, USA).

### Luciferase reporter assay

To detect the bind ability between PCGEM1 (SOX11) and miR-590-3p, wide type full-length sequences of PCGEM1 (SOX11) and the mutant-type PCGEM1 (SOX11) were cloned into the firefly luciferase gene reporter vector, pmirGLO (Promega, Madison, WI, USA). The plasmid was synthesized by Invitrogen. The pmirGLO-PCGEM1(SOX11)-Wt or pmirGLO-PCGEM1 (SOX11)-Mut was co-transfected with miR-590-3p mimics (inhibitor) or NC mimics (inhibitor) (RiboBio, Guangzhou, China) into HEK293T cells. After 48-hour of transfection, the luciferase assay was performed with the dual-luciferase reporter assay system kit (Promega) according to the manufacturer’s guidance.

### RNA pull down

Biotinylated PCGEM1 (PCGEM1 probe-biotin) and negative control (PCGEM1 probe-no biotin) (Sangon, Shanghai, China) were co-transfected into NSCLC cells. Cells were lysed and collected after transfection. After incubation with Dynabeads M-280 Streptavidin (Invitrogen) for 10 min, the bound RNAs were subjected to RT-qPCR for quantification and analysis.

### RNA immunoprecipitation (RIP) assay

RIP assay was performed with an EZ-Magna RIP RNA-Binding Protein Immunoprecipitation Kit (Millipore, Billerica, MA) based on the manufacturer’s guidance. The RIPA lysis buffer containing protease inhibitor cocktail and RNase inhibitor was made to lyse cells. The cells were incubated with RIPA buffer containing magnetic beads coated with Ago2 antibodies (Millipore, Billerica, MA). IgG group was utilized as a negative control group. After incubation at 4 °C for 2 h, the coprecipitated RNA was eluted from the beads and measured by NanoDrop spectrophotometer (Thermo Fisher Scientific, Shanghai, China).

### Nude mice model

A total of 15 BALB/c nude mice at the age of 4 ~ 5 weeks of both sexes were purchased from the Kunming Institute of Zoology, Chinese Academy of Sciences and were raised in a specific pathogen-free environment. Animal experiments were approved by the animal ethics committee of the China-Japan Friendship Hospital. A549 cells (5 × 10^6^) stably infected with lentiviruses containing sh-PCGEM1 or SOX11 were suspended in serum-free DMEM medium and then inoculated into left armpit of mice (5 mice in each group) to establish heterotopic transplanted tumor models of NSCLC. Mice were grouped as follows: (1) the sh-NC group; (2) the sh-PCGEM1 group; (3) the sh-PCGEM1 + SOX11 group. Tumor growth was recorded every 5 days by measuring tumor length and width using a vernier caliper. The tumor volume was calculated with the formula volume = (length × width^2^)/2. At day 25 after inoculation, the mice were euthanized and the tumor tissues to collected for weighing.

### Statistical Analysis

The data acquired were displayed as mean ± standard deviation. Data analysis was conducted with SPSS 20.0 software (SPSS Inc., Chicago, IL, USA). All experiments were repeated three times. One-way ANOVA was conducted for comparison of differences among 3 groups, and Student’s t test was conducted for comparison between 2 groups. Moreover, gene expression correlation was analyzed by Spearman’s correlation analysis. P < 0.05 represented statistically differential significance.

## Results

### PCGEM1 promoted NSCLC cell proliferation, migration, invasion and EMT process in vitro

We performed RT-qPCR analysis to testify PCGEM1 expression in NSCLC. As displayed in Fig. 1A, the expression of PCGEM1 showed significant upregulation in NSCLC tissues. Meanwhile, PCGEM1 expression was higher in NSCLC cells than in normal cells (Fig. 1B). To investigate possible biological role of PCGEM1 in proliferation, migration, and invasion of NSCLC cells, loss-of-function experiments were conducted. We first knocked down PCGEM1 expression with sh-PCGEM1#1 or sh-PCGEM1#2 and then detected the efficiency of PCGEM1 knockdown. We found that PCGEM1 expression in NSCLC cells in sh-PCGEM1#1/2 groups was reduced compared with that in the sh-NC group. Moreover, we found that PCGEM1 silencing attenuated cell viability (Fig. 1D). PCGEM1 knockdown had an inhibitory effect on NSCLC colony formation ability (Fig. 1E). Furthermore, PCGEM1 knockdown inhibited cell migratory and invasive capacities of NSCLC cells (Fig. 1F, G). In addition, according to western blot results, expression of epithelial marker, E-cadherin, showed significant upregulation, while expression of mesenchymal marker, N-cadherin, showed downregulation under silencing PCGEM1 in NSCLC cells (Fig. 1H).

**Fig. 1:** PCGEM1 facilitated cell proliferation and migration in NSCLC. **A** PCGEM1 levels in NSCLC tissues and normal tissues were tested with RT-qPCR. **B** RT-qPCR examined PCGEM1 levels in 4 NSCLC cells and BEAS-2B cells. **C** Silencing efficacy of PCGEM1 in NSCLC cells was tested via RT-qPCR. **D** Cell viability under sh-PCGEM1#1/2 was detected via CCK-8. **E** Colony formation experiment confirmed cell proliferative ability after silencing PCGEM1. **F**, **G** Cell migration and invasion upon PCGEM1 knockdown were measured through transwell assays. **H** Levels of EMT markers were assessed with western blot analysis after silencing PCGEM1. *p < 0.05, **p < 0.01

### MiR-590-3p was the downstream gene of PCGEM1

More and more evidence has revealed that lncRNAs contain sequences complementary to miRNAs, thereby regulating expression of miRNAs. Hence, we supposed that PCGEM1 exerts a carcinogenic effect via functioning as a ceRNA in NSCLC cells. Top five potential downstream miRNAs of PCGEM1 were predicted from DIANA database (Fig. 2A). Next, RNA pull down results indicated that miR-590-3p or miR-3157-5p could bind with PCGEM1, while miR-548ar-3p, miR-548az-3p, miR-548e-3p was not significantly pulled down by PCGEM1 probe-biotin (Fig. 2B). Additionally, miR-590-3p expression presented a significant decline in 4 NSCLC cells compared with that in control BEAS-2B cell line (Fig. 2C). Therefore, miR-590-3p could be identified as downstream of PCGEM1. Furthermore, miR-590-3p showed significantly downregulated expression in NSCLC tissues rather than in normal tissues (Fig. 2D). Moreover, miR-590-3p expression in NSCLC cells was increased under treatment of miR-590-3p mimics and decreased under treatment of miR-590-3p inhibitor (Fig. 2E). Binding sequence of PCGEM1 and miR-590-3p was predicted based on the DIANA online tool (Fig. 2F). The result of luciferase reporter experiment suggested that wide-type PCGEM1 luciferase activity was decreased by upregulated miR-590-3p compared to the control group, whereas luciferase activity of PCGEM1-Mut presented no significant change under the same condition (Fig. 2G). Additionally, we found the negative expression correlation of PCGEM1 and miR-590-3p in NSCLC tissues (Fig. 2H).

**Fig. 2:** MiR-590-3p was sponged by PCGEM1. **A** The putative downstream miRNAs of PCGEM1 was predicted using DIANA database. **B** RNA pull down assay revealed the binding between the predicted 5 miRNAs and PCGEM1. **C** Expression of two candidate targets in NSCLC cells and BEAS-2B cells were confirmed by RT-qPCR. **D** RT-qPCR validated miR-590-3p expression in NSCLC and adjacent tissues. **E** The transfection efficiencies of miR-590-3p mimics or miR-590-3p inhibitor in NSCLC cells were tested by RT-qPCR. **F** Predicted binding fragment of miR-590-3p and PCGEM1 was predicted from DIANA database. **G** The binding between PCGEM1 and miR-590-3p in NSCLC cells was further verified though luciferase reporter assay. **H** Expression correlation of PCGEM1 and miR-590-3p in NSCLC tissues was determined by Spearman analysis. *p < 0.05, **p < 0.01

### The carcinogenic effect of PCGEM1 on NSCLC was reversed by miR-590-3p

We wondered whether miR-590-3p reverses PCGEM1-mediated effects on NSCLC cells and conducted some rescue experiments. First, the miR-590-3p inhibitor and sh-PCGEM1#1 were co-transfected into A549 cells. MiR-590-3p downregulation counteracted the inhibitive function of PCGEM1 silencing on viability of A549 cells (Fig. 3A). Moreover, miR-590-3p knockdown rescued the inhibited cell proliferative ability of A549 cells caused by PCGEM1 knockdown (Fig. 3B). In addition, miR-590-3p inhibitor rescued the suppressed migrative and invasive abilities of A549 cells mediated by PCGEM1 silencing (Fig. 3C). Furthermore, western blot results revealed that miR-590-3p downregulation counteracted the PCGEM1 silencing-mediated suppression on the EMT process (Fig. 3D).

**Fig. 3:** The effect of PCGEM1 on NSCLC was counteracted by miR-590-3p. **A** CCK-8 assay testified viability of NSCLC cells after co-transfection. **B** Colony formation assay measured proliferative capability of NSCLC cells after indicated transfection. **C** Cell migration and invasion in each group were respectively assessed by transwell assay. **D** Western blot analysis was applied to assess levels of EMT markers in each group. *p < 0.05

### SOX11 was targeted by miR-590-3p

To confirm ceRNA supposition, we searched the potential targets of miR-590-3p. There are seven mRNAs as putative miR-590-3p targets (predicted score: 1) based on bioinformatics tool (DIANA) (Fig. 4A). Next, expression levels of seven mRNAs under miR-590-3p overexpression or knockdown were testified through RT-qPCR. As a result, only SOX11 could be downregulated by miR-590-3p upregulation or upregulated by miR-590-3p downregulation (Fig. 4B). Thus, SOX11 was selected for the subsequent experiments. Moreover, the binding site of miR-590-3p and SOX11 was obtained from online prediction tool TargetScan (Fig. 4C). To validate binding ability of SOX11 and miR-590-3p, luciferase reporter experiment was conducted using SOX11-WT and SOX11-MUT plasmids. Results indicated that wild-type SOX11 luciferase activity was declined under miR-590-3p mimics and was increased under miR-590-3p inhibitor compared to the control group, whereas luciferase activity of SOX11-Mut presented no significant change (Fig. 4D). Furthermore, as illustrated in Fig. 4E, both SOX11 and miR-590-3p demonstrated significant enrichment in Ago2-conjugated beads rather than in control IgG group. In addition, compared to the sh-NC group, sh-PCGEM1#1 reduced SOX11 expression (Fig. 4F). In addition, SOX11 expression showed significant upregulation in NSCLC cells compared to BEAS-2B cells (Fig. 4G). SOX11 expression was also upregulated in NSCLC tissues compared to that in adjacent nontumor tissues (Fig. 4H). Spearman’s correlation analysis depicted that SOX11 expression was negatively correlated to miR-590-3p expression but positively correlated to PCGEM1 expression in NSCLC tissues (Fig. 4I, J).

**Fig. 4:** SOX11 was downstream of miR-590-3p. **A** Putative targets of miR-590-3p were obtained by DIANA database. **B** Expression levels of seven candidate targets were testified by RT-qPCR upon miR-590-3p overexpression or downregulation. **C** Predicted site of miR-590-3p on SOX11 was predicted with online tool TargetScan database. **D** Luciferase reporter assay validated binding relationship of SOX11 and miR-590-3p in NSCLC cells. **E** Relative enrichment of SOX11 and miR-590-3p in the Ago2 precipitated RISCs in NSCLC cells was further confirmed via RIP assay. **F** Effect of PCGEM1 knockdown on SOX11 expression in NSCLC cells was validated by RT-qPCR. **G** RT-qPCR examined PCGEM1 expression in NSCLC cells and BEAS-2B cells. **H** RT-qPCR examined PCGEM1 expression in NSCLC tissues and corresponding nontumor tissues. **I**, **J** Correlation between SOX11 expression and miR-590-3p (PCGEM1) expression in NSCLC tissues was determined by Spearman’s correlation analysis. *p < 0.05, **p < 0.01.

### PCGEM1 functioned as an oncogene in NSCLC via modulating SOX11 expression

We conducted some rescue experiments to testify the rescue effects of SOX11 on NSCLC cell functions. First, we transfected NSCLC cell lines with pcDNA3.1 or pcDNA3.1/SOX11 and SOX11 expression was elevated by pcDNA3.1/SOX11 (Fig. 5A). Inhibitory effect of PCGEM1 downregulation on cell viability of NSCLC was countervailed by SOX11 upregulation (Fig. 5B). Moreover, cell proliferation of NSCLC attenuated by PCGEM1 knockdown was reversed by SOX11 overexpression (Fig. 5C). In addition, upregulated SOX11 rescued the repressive function of PCGEM1 knockdown on migrative and invasive abilities of NSCLC cells (Fig. 5D). In addition, western blot analysis presented that PCGEM1 knockdown-mediated inhibition on the EMT process was counteracted under SOX11 overexpression (Fig. 5E). Further in vivo assays revealed that depletion of PCGEM1 suppressed xenograft tumor growth and weight and such effect was rescued by overexpression of SOX11 (Fig. 5F–H).

**Fig. 5:** PCGEM1 promoted proliferative and migrative abilities of NSCLC cells through upregulating SOX11 expression. **A** RT-qPCR measured SOX11 overexpression efficacy. **B** CCK-8 assay detected the viability of A549 cells under indicated transfection. **C** Proliferation of A549 cells in indicated transfection group was testified with colony formation experiment. **D** Cell migration and invasion in each group were assessed via transwell experiments. **E** Western blot analysis evaluated protein levels of EMT markers after indicated transfection. **F** Images of tumors dissected from the mice in the sh-NC, sh- PCGEM1, and sh-PCGEM1 + SOX11 group. **G**, **H** Tumor growth curve and tumor weight of mice in the sh-NC, sh- PCGEM1, and sh-PCGEM1 + SOX11 group. *p < 0.05, **p < 0.01

## Discussion

Recently, many studies have shown that PCGEM1 has an oncogenic effect on numerous cancers, including renal carcinoma [14], cervical cancer [15], and gastric cancer [17]. In this study, we first revealed that PCGEM1 was upregulated in NSCLC cells and tissues. Next, we performed loss-of-function assays to figure out the role of PCGEM1 in NSCLC. We found that PCGEM1 knockdown inhibited NSCLC cell viability, proliferation, migration, and invasion. Therefore, our data revealed that PCGEM1 served as an oncogene in NSCLC (Additional file 1).

Competitive endogenous RNA (ceRNA) network is a common post-transcriptionally regulatory mechanism and refers to that lncRNAs compete with mRNAs to bind with miRNAs to free the suppressive effects of miRNAs on mRNAs [18, 19]. We explored whether PCGEM1 functions as a ceRNA to upregulate certain mRNA in NSCLC. MiR-590-3p was verified as the downstream gene of PCGEM1 through a series of mechanism assays. Previous reports revealed that miR-590-3p has a tumor inhibitive impact on certain cancers, including triple-negative breast cancer [20], prostate cancer [21], gastric cancer [22]. However, biological function of miR-590-3p in NSCLC has not been studied yet. In our study, mechanistical experiments verified the interaction of PCGEM1 and miR-590-3p, and there was a negative expression correlation between these two genes. In brief, PCGEM1 could bind with miR-590-3p. Furthermore, more rescue assays verified that miR-590-3p knockdown could recover inhibitory influence of silenced PCGEM1 on NSCLC viability, proliferation, migration, and invasion.

Mechanistically, we verified that SOX11 was a target of miR-590-3p. Moreover, SOX11 was reported as an oncogene in bladder cancer [23], lymphoma [24] and ductal carcinoma [25]. RT-qPCR analysis in our report indicated that SOX11 was upregulated in NSCLC tissues and cells. We found that SOX11 expression was negatively correlated to miR-590-3p expression, while positively correlated to PCGEM1 expression. In summary, PCGEM1 upregulated SOX11 expression through sponging miR-590-3p. Moreover, results of rescue experiments revealed that the PCGEM1 knockdown-mediated inhibition on proliferation and migration of NSCLC cells could be reversed under SOX11 upregulation.

## Conclusions

To sum up, our data initially proved the upregulated expression of PCGEM1, SOX11 and downregulated expression of miR-590-3p in NSCLC cells and tissues. LncRNA PCGEM1 contributed to cell proliferation, migration, invasion and EMT process in NSCLC via modulating the miR-590-3p/SOX11 axis. The findings indicated that PCGEM1 could offer a new thought for treatment of NSCLC.

## Supplementary Information

**Additional file 1:** Original uncropped western blot gels.

## Data Availability

All data from this study are available in this published article.

## Abbreviations

NSCLC: Non-small cell lung cancer
LncRNAs: Long non-coding RNAs
SOX11: SRY-box transcription factor 11
MiRNAs: microRNAs.
RIP: RNA immunoprecipitation
CeRNA: Competitive endogenous RNA
